The article "Effects of Albumin Supplements on In-Hospital Mortality in Patients with Sepsis or Septic Shock: A Systemic Review and Meta-Analysis" was retracted in 2023. Reasons: unreliable results or conclusions; concerns about the data; concerns about the peer review; concerns about the citations.

# Effects of Albumin Supplements on In-Hospital Mortality in Patients with Sepsis or Septic Shock: A Systemic Review and Meta-Analysis

**DOI:** 10.1155/2022/2384730

**Published:** 2022-10-10

**Authors:** Pei Liu, Deyuan Zhi, Yajun Wang, Jin Lin, Meng Zhang, Meili Duan

**Affiliations:** Department of Critical Care Medicine, Beijing Friendship Hospital, Capital Medical University, Beijing, China

## Abstract

**Objective:**

To explore the clinical effects of albumin supplements on the basis of crystalloid solution in patients with sepsis or septic shock.

**Methods:**

The online databases including PubMed, Web of Science, Cochrane Library, and EMBASE were comprehensively searched from inception to June 28, 2021, with the keywords including “albumin,” “sepsis,” or “septic shock.” Retrospective cohort (RC) and randomized controlled trials (RCT) were included for analysis. Two authors independently searched and analyzed the literature. The in-hospital mortality at 7 days and 28 days, duration of mechanical ventilation, renal replacement therapy, length of ICU stay, and length of hospital stay were compared between patients with albumin supplements and crystalloid solution and those with crystalloid alone.

**Results:**

A total of 10 studies with 6463 patients were eventually included for meta-analysis. The in-hospital mortality of patients at 7 days (OR = 1.00, 95% CI: 0.81–1.23) and 28 days (OR = 1.02, 95% CI: 0.91–1.13) did not show a significant difference between the two groups of patients. Also, the pooled results demonstrated no significant differences in duration of mechanical ventilation (OR = 0.29, 95% CI: −0.05–0.63), renal replacement therapy (WMD = 1.15, 95% CI: 0.98–1.35), length of ICU stay (WMD = −0.07, 95% CI: −0.62–0.48), and length of hospital stay (WMD = −0.09, 95% CI: −0.70–0.52) between patients receiving albumin plus crystalloid solution and those with crystalloid solution alone.

**Conclusion:**

Albumin supplements on the basis of crystalloid solution did not improve the 7-day and 28-dayin-hospital mortality in patients with sepsis or septic shock compared with those with crystalloid solution alone.

## 1. Introduction

Severe infections often lead to septic shock, which refers to sepsis syndrome with shock caused by microorganisms and toxins or metabolites [1]. Toxins and cell wall products in the lesions of septic shock patients invade the blood circulation, directly activate the host cells and humoral systems, synthesize and release endogenous mediators and cytokines, and act on important organs, tissues, and systems of the body, thereby seriously affecting the perfusion of these organs [2]. Severe infection-induced septic shock always leads to ischemia and hypoxia in tissue cells, increases the risk of metabolic disorders and dysfunctions of important organs and tissues, and even severe multiorgan failure in a small number of patients [3]. In clinical practice, it is difficult to treat septic shock. Since there is a high risk of death, most patients have a poor prognosis. In addition to actively controlling infection, the treatment of septic shock should also include supplementation of blood volume, correction of acidosis, adjustment of vasomotor function, elimination of blood cell aggregation, prevention of circulatory stasis, and maintenance of important organ functions [4]. The most important issue for successful treatment is to restore the normal blood perfusion, internal environment, and metabolism of the vital organs of the body [5].

The article "Effects of Albumin Supplements on In-Hospital Mortality in Patients with Sepsis or Septic Shock: A Systemic Review and Meta-Analysis" was retracted in 2023. Reasons: unreliable results or conclusions; concerns about the data; concerns about the peer review; concerns about the citations.

Adequate fluid resuscitation in the early stage to maintain effective vascular volume and tissue perfusion can significantly improve the prognosis of patients with sepsis. Crystalloid solutions are frequently used for fluid resuscitation in critically ill patients due to their advantages such as effectiveness and low cost and availability. The crystalloid solution is composed of small molecules such as sodium ions and chloride. However, a large amount of crystalloid solution may cause adverse reactions such as hypernatremia, hyperchloremia, and acidosis, which may negatively affect the coagulation function, renal function, gastrointestinal function, and respiratory function of patients [6]. Human albumin is a nonglycosylated, small molecular weight, negatively charged serum protein with a high level in plasma, accounting for about 55% of plasma proteins. It is completely synthesized by the liver and has a long half-life of about 20 days [7]. As the main substance to maintain plasma colloid osmotic pressure, albumin is the carrier of many endogenous and exogenous substances. It has anti-inflammatory and antioxidant effects, can remove active oxygen groups and nitrogen groups in the body, and also maintains acid-base balance [8]. The relative molecular mass of albumin is large, which can effectively maintain the expansion of intravascular fluid for a long time. Compared with crystalloid solution, albumin may be superior to increasing colloid osmotic pressure and central venous pressure [9]. However, the use of albumin for the treatment of sepsis is still controversial at present.

In order to investigate the effects of albumin supplements in patients with sepsis, we performed this systemic review and meta-analysis to summarize and analyze the currently available evidence on the albumin in the treatment of sepsis. We hope to provide evidence-based medical data for optimizing the treatment strategy for critically ill patients with sepsis.

The article "Effects of Albumin Supplements on In-Hospital Mortality in Patients with Sepsis or Septic Shock: A Systemic Review and Meta-Analysis" was retracted in 2023. Reasons: unreliable results or conclusions; concerns about the data; concerns about the peer review; concerns about the citations.

## 2. Materials and Methods

### 2.1. Search Strategy and Literature Inclusion

We performed this systemic review and meta-analysis strictly in accordance with the requirements in Preferred Reporting Items for Systematic Reviews and Meta-Analyses (PRISMA) [10]. The online databases including PubMed, Web of Science, Cochrane Library, and EMBASE were comprehensively searched with the keywords including “albumin,” “sepsis,” or “septic shock.” The retrieved literature was published from inception to June 28, 2021. Two authors independently searched and included the studies. All articles were firstly reviewed by title and abstract, and the potentially eligible studies were further reviewed by reading the full text. A study was eventually included if the inclusion and exclusion criteria were met. If different opinions occurred for the article, a senior researcher in the field was asked for further evaluation and determination of the inclusion or exclusion of the article.

### 2.2. Inclusion and Exclusion Criteria

Studies meeting the following criteria were eligible for inclusion: (1) the study design was prospective; (2) the study population was adult patients with sepsis or septic shock; (3) the intervention: patients in the study group were given albumin on the basis of crystalloid solution for fluid resuscitation, and patients in the control group were only given crystalloid solution for fluid resuscitation; (4) main outcome was in-hospital mortality at 7 days, 28 days or 90 days. Studies with one of the following criteria were excluded: (1) reduplicated studies; (2) data were inadequate; (3) case reports, reviews, and conference abstracts.

### 2.3. Data Extraction

For each eligible study, the authors, study periods, age of patients, study design, diseases, sample size, albumin concentration, crystalloid, follow-up, and outcomes were collected and recorded for further analysis.

### 2.4. Main Outcomes

The main outcomes in this systemic review and meta-analysis were in-hospital mortality of patients at 7 days, 28 days, or 90 days. Duration of mechanical ventilation, length of intensive care unit (ICU) stay and length of hospital stay, and renal replacement therapy were also collected and investigated.

### 2.5. Evaluation of Study Quality

The revised Cochrane risk of bias tool (RoB2.0) was used for evaluating the quality of included studies. The risk of bias was shown in Table 1 for details. In order to assess the publication bias, funnel plots were drawn and visually evaluated the symmetry of the plots.

### 2.6. Statistical Analyses

In this study, Stata 14.0 and Review Manager 5.0 software were applied for analysis. The ORs and 95% confidence interval (95% CI) were used to compare the effect of albumin in addition to the crystalloid solution on in-hospital mortality at 7 days and 28 days, as well as renal replacement therapy between the two groups. Weighted mean difference (WMD) and 95% CI were used to compare the duration of mechanical ventilation, length of ICU stay, and length of hospital stay between patients with albumin supplements and crystalloid solution and those with crystalloid alone. In order to evaluate the heterogeneity among different studies, we used the Cochran *Q* test and *I*^2^ statistic for determining the type of effect model used. If *P* < 0.01 in the *Q* test or *I*^2^ statistic > 50%, a random-effect model was used since there was significant heterogeneity. Otherwise, a fixed-effect model was adopted.

The article "Effects of Albumin Supplements on In-Hospital Mortality in Patients with Sepsis or Septic Shock: A Systemic Review and Meta-Analysis" was retracted in 2023. Reasons: unreliable results or conclusions; concerns about the data; concerns about the peer review; concerns about the citations.

## 3. Results

### 3.1. Study Characteristics

According to the aforementioned keywords used in searching the literature, a total of 201 potentially relevant articles were preliminarily obtained. After reviewing the title and abstract of these articles, 175 irrelevant articles were excluded. For the remaining 26 articles, there were 3 articles with repeated research, 4 articles with incomplete data for meta-analysis, 6 articles of reviews or systemic reviews, and 3 irrelevant studies. Eventually, ten studies [8, 11–19], which were published between 2004 and 2021, were included for further analysis. The characteristics of these studies were shown in Table 1 for details. A total of 6463 patients were included, in which 2979 patients (46.1%) in the study group received albumin supplement and crystalloid solution for fluid resuscitation, and 3484 patients (53.9%) in the control group were given crystalloid solution such as saline alone for resuscitation. (see Table 2).

### 3.2. Effect of Albumin Supplements on In-Hospital Mortality

In order to evaluate the effect of albumin supplements on the in-hospital mortality of patients with sepsis or septic shock, we summarized the relevant data by meta-analysis. Three studies [15, 17, 18] assessed the mortality of patients at 7 days, and no statistically significant difference was detected between the two groups of patients according to the results of pooled analysis (Figure 1, OR = 1.00, 95% CI: 0.81–1.23). Nine studies [8, 11–17, 19] explored the mortality of patients at 28 days, and the pooled result showed that the mortality was not statistically different between patients with albumin supplements and those without supplements (Figure 2, OR = 1.02, 95% CI: 0.91–1.13). Funnel plots did not find significant publication bias of these studies (Supplementary Figures 1 and 2). Further subgroup analysis with 4 studies [11–13, 16] for patients with septic shock showed that albumin supplements did not affect the 28-day mortality of these patients (Supplementary Figure 3, OR = 1.06, 95% CI: 0.88–1.28).

The article "Effects of Albumin Supplements on In-Hospital Mortality in Patients with Sepsis or Septic Shock: A Systemic Review and Meta-Analysis" was retracted in 2023. Reasons: unreliable results or conclusions; concerns about the data; concerns about the peer review; concerns about the citations.

### 3.3. Effect of Albumin Supplement on Duration of Mechanical Ventilation, Renal Replacement Therapy, Length of ICU Stay, and Hospital Stay

As for other outcomes including duration of mechanical ventilation, renal replacement therapy, length of ICU stay, and length of hospital stay, a total of 3 studies [8, 15, 16], 4 studies [8, 15–17], 4 studies [8, 15–17], and 4 studies [8, 15–17], respectively, investigated the effects of albumin supplement on these parameters. Interestingly, the pooled results did not show significant differences in the duration of mechanical ventilation (Figure 3, SMD = 0.29, 95% CI: −0.05–0.63), renal replacement therapy (Figure 4, OR = 1.15, 95% CI: 0.98–1.35), length of ICU stay (Figure 5, WMD = −0.07, 95% CI: −0.62–0.48), and length of hospital stay (Figure 6, WMD = −0.09, 95% CI: −0.70–0.52) between patients receiving albumin plus crystalloid solution and those with crystalloid solution alone.

## 4. Discussion

In this study, we performed a systemic review and meta-analysis of the currently available literature on supplementation of albumin in addition to a crystalloid solution for the treatment of patients with sepsis. The pooled analysis did not find significant differences between the study group and control group in the 7-day mortality, 28-day mortality, duration of mechanical ventilation time, renal replacement therapy, length of ICU stay, and total hospital stay. These results indicate albumin and crystalloid as resuscitation fluids did not differ in clinical outcomes in adult patients with sepsis or septic shock, and there is no significant clinical benefit with the use of albumin. Our study provides new insights into the clinical decision-making on the selection of agents for fluid resuscitation in patients with sepsis.

Sepsis is a severe stage of infection, with high mortality and poor prognosis during hospitalization. Clinically, catecholamine vasoconstrictor drugs and fluid resuscitation are often given to patients with septic shock. However, when the body is in a state of persistent infection, the response of blood vessels to the catecholamine drugs is reduced, and the treatment effect is limited. Early and effective fluid resuscitation is one of the most important widely used clinical treatment strategies. However, the selection of colloid or crystalloid as the resuscitation fluid has been controversial for a long time. Crystalloids mainly include various concentrations of sodium chloride solution, Ringer's solution, and equilibrium solution, while human albumin is a common colloidal solution preparation.

The article "Effects of Albumin Supplements on In-Hospital Mortality in Patients with Sepsis or Septic Shock: A Systemic Review and Meta-Analysis" was retracted in 2023. Reasons: unreliable results or conclusions; concerns about the data; concerns about the peer review; concerns about the citations.

Albumin is a negatively charged, small molecular weight, nonglycosylated serum protein with functions including substance binding and transport, enzymatic activity, and antioxidation [20]. Albumin is mainly synthesized and secreted by hepatocytes in the liver, secreted into the sinusoids, and then enters the blood circulation. The half-life of albumin is relatively long, for generally 17–20 days, after which degraded in muscle, liver, and kidney [21]. Albumin can bind a variety of endogenous and exogenous compounds, such as fatty acids, metal ions, metabolites, and drugs, which suggest that albumin may be used for the treatment of septic shock [22]. The occurrence and development of septic shock are affected by many factors, and it is a pathophysiological process in which many cytokines participate together. Aerobic metabolism is a normal physiological process of the body, but for patients with septic shock, aerobic metabolism occurs during treatment, and some of the intermediate products may cause the accumulation of toxic substances, such as reactive oxygen species and reactive nitrogen species, causing cell damage and dysfunction, which is also one of the main causes of death in patients with septic shock during treatment [23] Theoretically, albumin can remove a variety of reactive oxygen species and reactive nitrogen produced by different ways, reduce the accumulation of toxic substances in patients, reduce cell damage and the risk of organ dysfunction [24]. In addition, albumin can combine with nitric oxide, bilirubin, and other substances with antioxidant effects to play an antioxidant role; meanwhile, many metal ions such as copper and iron can combine with albumin to catalyze and reduce the body's peroxidative damage [25]. In addition to albumin therapy, patients with septic shock will be treated with various other drugs during the treatment period. The cysteine binding mechanism on the amino acid sequence of albumin indicates that it may enhance the clinical efficacy of drugs in septic shock. However, our results in this study did not find significant differences in various clinical outcomes including 7-day and 28-day mortality, mechanical ventilation, renal replacement therapy, length of ICU stay, and hospital stay. Patients with septic shock did not benefit from the application of albumin. Therefore, more studies are needed to further confirm the significance of albumin administration in patients with sepsis.

Insufficiency of circulating blood volume is the main manifestation of infectious patients. It is mostly caused by the large opening of the venous vascular bed and the decrease in peripheral vascular resistance, resulting in abnormal distribution of blood flow. Meanwhile, severe leakage of capillaries can lead to severe hypoperfusion. So, reasonable and effective fluid resuscitation is of great clinical importance for these critically ill patients [26]. A previous study found that when the perfusion pressure was severely insufficient, the body's compensatory ability cannot resist the occurrence of tissue edema, thereby further increasing the risk of tissue edema. The serious insufficiency of perfusion pressure will lead to pulmonary edema and increase the risk of in-hospital mortality [27]. Reasonably improving tissue hypoperfusion and relieving tissue ischemia and hypoxia is of great significance for improving patient prognosis and reducing the risk of death. The maintenance of colloid osmotic pressure has a positive significance in the treatment of septic shock [28]. The negative charge on the surface of albumin can attract sodium ions and play a role in retaining water. Also, albumin can maintain 70% to 80% of the colloidal osmotic pressure in plasma at normal levels [29]. Since the results of this study showed that albumin supplements did not improve the clinical prognosis of patients with sepsis, it is worth exploring the role of albumin on osmotic pressure in the conditions of sepsis.

The article "Effects of Albumin Supplements on In-Hospital Mortality in Patients with Sepsis or Septic Shock: A Systemic Review and Meta-Analysis" was retracted in 2023. Reasons: unreliable results or conclusions; concerns about the data; concerns about the peer review; concerns about the citations.

Most patients with septic shock are accompanied by severe organ dysfunction, and a small number of patients may be combined with multiple organ failures. The continuous decline of organ function is the key reason for the high risk of death in patients. Therefore, during the systemic treatment of septic patients, protection of the organ function, and prevention of the damage to the normal organ by sepsis is also the key to treatment [27]. Albumin is considered to be effective in improving blood perfusion of organs, inhibiting the occurrence of inflammatory reactions, and combining with drugs used in comprehensive treatment, thereby play a role in protecting the important organs. A previous study found that the combined use of human albumin and cefotaxime sodium can reduce the damage to the kidneys caused by other drugs during treatment, and greatly reduce the mortality rate of patients [30]. However, our results showed that the albumin supplement did not influence the renal replacement therapy in patients with sepsis, suggesting that albumin may act on other roles for the important organs. In addition, studies have found that in the process of shock and resuscitation in critically ill patients, the use of 25% human albumin can reduce damage to lung tissue by regulating the expression of inflammatory factors in endothelial cells, thereby reducing damage to lung tissue [31].

The article "Effects of Albumin Supplements on In-Hospital Mortality in Patients with Sepsis or Septic Shock: A Systemic Review and Meta-Analysis" was retracted in 2023. Reasons: unreliable results or conclusions; concerns about the data; concerns about the peer review; concerns about the citations.

Hypoalbuminemia is an independent risk factor for severe comorbidities and death in patients with septic shock [32]. Whether the role of human albumin in the treatment of hypoalbuminemia is reliable in septic shock has always been a hot topic of clinical debate [33]. A previous study found that the use of human albumin in critically ill patients did not affect the mortality rate, but for patients with septic shock and severe burn shock, the use of human albumin may increase the risk of death [30]. A study of 6997 critically ill patients compared 0.9% sodium chloride injection with human serum albumin for fluid resuscitation. The results showed that there was no statistically significant difference in mortality and treatment duration between the two groups [34]. Therefore, albumin and crystalloid have no difference in the prognosis of adult patients with sepsis and septic shock. In addition, when paying attention to the resuscitation effect of human albumin, it should also be fully considered that albumin may increase medical costs and the risk of transfusion of blood products.

### 4.1. Limitations

This study has some limitations. First, the number of eligible studies is relatively small, especially for those investigating the 7-dayin-hospital mortality, duration of mechanical ventilation, renal replacement therapy, length of ICU stay, and length of hospital stay. Second, the duration of follow-up of patients is relatively short, so the results of this study are limited to short-term prognosis. In the future, more randomized controlled studies (RCTs) with long-termfollow-ups are needed to further explore the role of albumin supplements in these critically ill patients. Meanwhile, different evidence weights should be paid special attention to when both RCT and non-RCT studies (NRS) were included for analysis [35]. Third, since the concentrations of albumin used in different studies are varied, it inevitably causes a certain bias in the results. Besides, the subgroup/sensitivity analysis restricting to those with low albumin levels can be performed to exhibit the effect of albumin supplements in patients with low albumin levels. More strict and unified RCTs may further confirm the conclusions in this study.

## 5. Conclusion

In conclusion, albumin supplements on the basis of crystalloid solution did not improve the 7-day and 28-dayin-hospital mortality in patients with sepsis or septic shock compared with those with crystalloid solution alone. Also, albumin did not affect the duration of mechanical ventilation, renal replacement therapy, length of ICU stay, and length of hospital stay in these patients.

The article "Effects of Albumin Supplements on In-Hospital Mortality in Patients with Sepsis or Septic Shock: A Systemic Review and Meta-Analysis" was retracted in 2023. Reasons: unreliable results or conclusions; concerns about the data; concerns about the peer review; concerns about the citations.

## Figures and Tables

**Figure 1:** Forest plot of odds ratio and 95% confidence interval on 7-dayin-hospital mortality of included studies.

**Figure 2:** Forest plot of odds ratio and 95% confidence interval on 28-dayin-hospital mortality of included studies.

**Figure 3:** Forest plot of weighted mean difference and 95% confidence interval on the duration of mechanical ventilation of included studies.

**Figure 4:** Forest plot of odds ratio and 95% confidence interval on renal replacement therapy of included studies.

**Figure 5:** Forest plot of weighted mean difference and 95% confidence interval on length of ICU stay of included studies.

**Figure 6:** Forest plot of weighted mean difference and 95% confidence interval on length of hospital stay of included studies.

**Table 1:** Baseline characteristics of included studies.

Study	Study period	Age median (IQR)	Study type	Patients	Sample size (study/ control)	Albumin (%)	Crystalloid	Follow-up	Outcome (study vs. control, %)	Risk
Chou et al	2009	N/A	RC	Sepsis	133 (52/81)	25% albumin	N/A	28-day mortality	48.1% (25/52) vs. 51.9% (42/81)	*M*
Annane et al	2013	Study: 63 (50–76) Control: 63 (50–75)	RCT	Sepsis	616 (59/557)	4%, 5%, 20% or 25% albumin	Isotonic or hypertonic saline	28-day and 90-day mortality	28-day: 32.2% (19/59) vs. 28.2% (157/557) 90-day: 37.3% (22/59) vs. 35.4% (197/557)	*L*
Park et al	2019	Study: 62 (51–70) Control: 61 (52–70)	RCT	Sepsis and Septic shock	360 (180/180)	4% albumin	Lactated Ringer's	7-day and 28-day mortality	7-day: 25.6% (46/180) vs. 22.2% (40/180) 28-day: 53.3% (96/180) vs. 46.1% (83/180)	*L*
Caironi et al	2014	Study: 70 (57–77) Control: 69 (59–77)	RCT	Sepsis and Septic shock	1810 (903/907)	20% albumin	N/A	28-day and 90-day mortality	28-day: 31.8% (285/895) vs. 32.0% (288/900) 90-day: 41.1% (365/888) vs. 43.6% (389/893)	*L*
Finfer et al	2011	Study: 60.5 ± 17.2 Control: 61.0 ± 17.1	RCT	Sepsis and Septic shock	1218 (603/615)	4% albumin	0.9% sodium chloride	28-day mortality	30.7% (185/603) vs. 35.3% (2174/615)	*L*
Liu et al	2021	Study: 67 (56–77) Control: 67 (54–77)	RC	Sepsis and Septic shock	835 (286/549)	5% or 20% albumin	N/A	28-day mortality	35.7% (102/286) vs. 31.7% (174/549)	*M*
Alexander et al	2021	Study: 59 (51–67) Control: 59 (50–68)	RC	Septic shock	360 (335/335)	25% albumin	N/A	28-day mortality	46.9% (157/335) vs. 44.8% (150/335)	*M*
Charpentier et al	2011	N/A	RCT	Septic shock	792 (399/393)	20% albumin	0.9% sodium chloride	28-day mortality	24.1% (96/399) vs. 26.2% (103/393)	*L*
Veneman et al	2004	N/A	RCT	Sepsis	31 (8/25)	20% albumin	0.9% sodium chloride	28-day mortality	62.5% (5/8) vs. 56.0% (14/25)	*H*
Philips et al	2021	Study: 49.4 ± 12.1 Control: 48.2 ± 10.6	RCT	Sepsis and Septic shock	308 (154/154)	5% albumin	0.9% sodium chloride	7-day mortality	43.5% (87/154) vs. 38.3% (95/154)	*M*

IQR: interquartile range; RC: retrospective cohort; RCT: randomized controlled trials; *M*: moderate risk; *L*: low risk; *H*: high risk.

The article "Effects of Albumin Supplements on In-Hospital Mortality in Patients with Sepsis or Septic Shock: A Systemic Review and Meta-Analysis" was retracted in 2023. Reasons: unreliable results or conclusions; concerns about the data; concerns about the peer review; concerns about the citations.

**Table 2:** Subgroup analysis for the effects of albumin vs. crystalloid on 28-day mortality of sepsis and/or septic shock.

Subgroup analysis	Studies	Pooled results		Heterogeneity	
		Effect size (95% CI)	*P* value	*I * ^2^	*P* value
Albumin concentration		OR			
4%-5%	4	1.01 (0.86–1.20)	0.861	54.0%	0.089
20%–25%	5	1.002 (0.88–1.18)	0.798	0%	0.461
Sample size		OR			
>650	5	0.99 (0.88–1.11)	0.834	35.3%	0.186
≤650	4	1.23 (0.92–1.66)	0.164	0%	0.555
Study type		OR			
RCT	6	0.96 (0.85–1.10)	0.576	27.7%	0.227
Retrospective study	3	1.17 (0.95–1.43)	0.139	0%	0.668

## Data Availability

The data used to support the findings of this study are included within the article.

## Supplementary Materials

Supplementary Materials Supplementary Figure 1. Funnel plot of publication bias of included studies investigating the 28-dayin-hospital mortality. Supplementary Figure 2. Begg's funnel plot of publication bias of included studies investigating the 28-dayin-hospital mortality. Supplementary Figure 3. Forest plot of odds ratio and 95% confidence interval on 28-dayin-hospital mortality of patients with septic shock.
